# circCNN2 Accelerates Cell Proliferation and Invasion in Lung Squamous Cell Carcinoma via Regulating miR-184/E2F1 and Activating MAPK Signaling Pathway

**DOI:** 10.1155/2022/6329097

**Published:** 2022-08-16

**Authors:** Shan Hu, Peng Cao, Kangle Kong, Peng Han, Jiaqi Yue, Yu Deng, Fan Li, Bo Zhao

**Affiliations:** Department of Thoracic Surgery, Tongji Hospital, Tongji Medical College, Huazhong University of Science and Technology, Wuhan 430030, China

## Abstract

Circular RNAs (circRNAs) have been demonstrated as potential biomarkers for the diagnosis and treatment of human diseases. Previous studies have unveiled the carcinogenic role of circRNA_102399 (circCNN2) in lung cancer. Through the UALCAN database, it was found that CNN2, the parent gene of circCNN2, was specifically highly expressed in human lung squamous cell carcinoma (LUSC) cells, but the regulatory mechanism of circCNN2 in LUSC is unclear. In this study, circCNN2 expression in LUSC cells was examined via RT-qPCR, and its effects on LUSC progression was verified through functional assays. The subcellular localization of circCNN2 was identified via FISH assay, and the underlying mechanism of circCNN2 on the activation of MAPK signaling pathway was determined through mechanism experiments. Results demonstrated that circCNN2 was upregulated in LUSC cells, and it promoted LUSC cell proliferation and invasion. Besides, circCNN2 acted as a competing endogenous RNA (ceRNA) to sponge miR-184 to upregulate E2F transcription factor 1 (E2F1) expression. Furthermore, it was verified that circCNN2 activated the generic mitogen-activated protein kinases (MAPK) signaling pathway through E2F1 and thus promoting LUSC progression. In a word, this study indicated that circCNN2 activated MAPK signaling pathway through the miR-184/E2F1 axis to promote proliferation and invasion of LUSC cells.

## 1. Introduction

Lung carcinoma represents one of the most common causes of cancer death in the world, and smoking is seen as the leading cause of lung cancer [1]. The major subtype of lung cancer is non-small-cell carcinoma (NSCLC) representing 80-90% of lung cancer cases, and NSCLC is further classified into two distinct types which include squamous cell carcinomas (LUSC) and adenocarcinomas (LUAD) from clinical, histological, genetic, and molecular perspectives [2]. Despite plenty of progresses made in LUSC treatment, it remains to be a highly metastatic disease associated with poor clinical prognosis [3]. Therefore, it is important to explore more potential biomarkers as well as molecular mechanisms so as to provide effective therapeutic options for the treatment of LUSC.

Circular RNAs (circRNAs) represent noncoding RNAs which are covalently closed molecules generated from back-splicing [4]. They are characterized by a covalently closed loop structure and have been reported to play as both tumor promoters and tumor suppressors in the regulation of lung cancer. For example, circular RNA 100146 and circSATB2 have been elucidated to promote NSCLC development [5, 6]. However, the detailed mechanism of circRNAs in LUSC progression is largely unknown [7]. Experimental data from early study unveiled that circRNA_102399 (circCNN2) was upregulated in lung cancer, and it promoted lung cancer development. In this study, we found through the UALCAN database that the parent gene of circCNN2, namely, CNN2, was with high expression in LUSC tumor samples. Therefore, we chose to conduct an in-depth study on the regulatory mechanism of circCNN2 on LUSC progression.

Emerging evidences have elucidated the role of circRNAs as ceRNAs in a broad range of cancers. For example, circHIPK3 promotes colorectal cancer growth and metastasis by sponging miR-7 [8], circRNA-104718 acts as a ceRNA and promotes hepatocellular carcinoma progression through the microRNA-218-5p/TXNDC5 signaling pathway [9]. The circTP63/FOXM1/miR-873-3p axis is identified to facilitate LUSC progression [10]. circTIMELESS regulates LUSC cell proliferation and invasion via the miR-136-5p/ROCK1 axis [11]. In this study, the ceRNA network of circCNN2/miR-184/E2F1 was identified in LUSC cells and related assays were carried out to testify its impact on LUSC progression.

The MAPK signaling pathway has been reported to be associated with cell proliferation, migration, and apoptosis [12–14]. In LUSC, fibroblast-derived exosomal microRNA-369 promotes migration and invasion of LUSC cells via the MAPK signaling pathway [15]. In this study, we also designed related assays to verify the interaction between circCNN2 and MAPK signaling in LUSC development.

In a word, we aimed to explore the regulatory function of circCNN2 in the progression of LUSC cells and to further verify the underlying mechanism of circCNN2 on the activation of the MAPK signaling pathway.

## 2. Materials and Methods

### 2.1. Cell Lines

Human LUSC cell lines SK-MES-1 (HTB-67), H1703 (CRL-2073), H226 (CRL-5826), H520 (HTB-182), and the normal human bronchial epithelial Beas-2B cell line (CRL-9609) were obtained from American Type Culture Collection (ATCC, Manassas, VA, USA). SK-MES-1 and Beas-2B cells were cultured in DMEM (12100046, Gibco, USA) while H1703, H226, and H520 cell lines were cultivated in RPMI 1640 medium (61870127, Gibco, USA). All the cells were supplemented with 10% fetal bovine serum (FBS; 10270-106, Gubco, USA) and 100× penicillin/streptomycin solution (SV30010, PERFEMIKER, Shanghai, China) in a humid incubator with 5% CO_2_ at 37°C.

### 2.2. Total RNA Extraction and Quantitative Real-Time Polymerase Chain Reaction (RT-qPCR)

The total RNA was extracted from cells by the TRIzol reagent (9108-1, Thermo Fisher, USA), and cDNA was synthesized by PrimerScript RT Reagent kit (Takara, Japan). RT-qPCR reaction was achieved with SYBR qPCR Master Mix (QR0100-1KT, Sigma-Aldrich, USA) in 20 *μ*l volume consisting of 2× SYBR Green Taq ReadyMix, 0.4 mM concentration of forward and reverse primers, and 10× PCR buffer. The qPCR reaction was performed under the condition of 95°C for 2 min, followed by 40 cycles of 95°C for 5 sec and 60°C for 15 sec, and finally 72°C for 10 sec. The relevant expression was determined by 2^-*ΔΔ*Ct^ method. In relevant assays, GAPDH and U6 were loading controls. All experiments were repeated for three times independently, and the results were presented in the form of mean ± standard deviation.

### 2.3. Cell Transfection

Specific shRNAs targeting circCNN2 (sh1/2/3-circCNN2) and E2F1 (sh1/2/3-E2F1), together with their negative control shRNAs (sh-NCs), were constructed to silence circCNN2 and E2F1 expressions. For the overexpression of E2F1, the whole sequences were synthesized and subcloned into pcDNA3.1 vector to construct pcDNA3.1-E2F1, with pcDNA3.1 empty vector as the negative control (NC). For the overexpression of miR-184, miR-184 mimics was used with mimics NC as the control, while for the silencing of miR-184, miR-184 inhibitor used with inhibitor NC as the control. In line with the supplier's protocols, transfections were conducted with Lipofectamine 2000 (11668019, Invitrogen, USA).

### 2.4. Cell Counting Kit-8 (CCK-8) Assay

Cell viability was evaluated with the application of CCK-8 kit (M4839, ABMOLE, USA) according to the manufacturer's guidelines. Transfected H1703 or H226 cells were seeded to 96-well plates adding 10 *μ*l of CCK-8 solution (Dojindo, Japan) at 37°C with 5% CO_2_ for 1 h. Absorbance was measured with the microplate reader (51119770DP, Thermo Fisher) at 450 nm.

### 2.5. Colony Formation Assay

800 cells were harvested after 48-hour transfection and were incubated in a 6-well plate for 14 days. The culture medium was discarded, and the cells were washed with PBS (C10010500BT, Gibco, USA). Cells were fixed with methanol solution for 15 minutes and then stained by crystal violet for 10 min at room temperature. Clones more than 50 cells were counted manually.

### 2.6. Transwell Assay

To evaluate the invasive ability of LUSC cells, cells were planted on the top of 24-well Transwell chambers coating Matrigel for invasion assay. The lower chambers were loaded with complete medium. Twenty-four hours later, cells in the upper layer were removed with caution by a cotton swab and then fixed in methanol solution for 15 min. Crystal violet was adopted to stain the membranes for 10 min, and the invaded cells were observed and counted under a microscope (10 × 10).

### 2.7. Western Blot Assay

Total protein extracted from LUSC cell lines was isolated by RIPA buffer, and after being separated through SDS-PAGE (P1200, Solarbio, Beijing, China), proteins were transferred to PVDF (T2234, Thermo Fisher, USA) membranes and blocked with 5% skim milk. The membranes were cultivated with primary antibodies overnight at 4°C, followed by being cultivated with secondary antibody for 1 h. After washing in TBST, the secondary antibodies were added and finally assayed by ECL Substrate. The quantitations of bands were determined by ImageJ software. The primary antibodies were listed as follows: anti-PCNA (ab29, 1 : 1000), anti-cyclin D1 (ab16663, 1 : 1000), anti-MMP2 (ab92536, 1 : 1000), anti-MMP9 (ab76003, 1 : 1000), anti-E2F1 (ab4070, 1 : 1000), anti-ASK1 (ab45178, 1 : 1000), anti-p38 (ab170099, 1 : 1000), anti-p-p38 (phospho T180 + Y182; ab4822, 1 : 1000), anti-Ki67 (ab15580, 1 : 1000), and the internal control GAPDH (ab181602, 1 : 1000). The above antibodies were all obtained from Abcam (UK).

### 2.8. RNA Immunoprecipitation (RIP) Assay

With the Imprint® RNA Immunoprecipitation Kit (RIP-12RXN, Sigma-Aldrich, USA), RIP assay in H1703 and H226 cells was achieved with the specific antibodies and normal control anti-IgG antibody. Lysates were obtained from LUSC cell lines using RIP lysis buffer. The lysis was incubated with the magnetic beads conjugated with the AGO2 antibody or IgG antibody (ab6789, Abcam, UK). The precipitated RNAs were analyzed by RT-qPCR.

### 2.9. RNA Pull Down Assay

With the application of Pierce RNA 3' End Biotinylation Kit (20160, Thermo Fisher, USA), RNA pull down assay was carried out in H1703 and H226 cells. Biotinylated circCNN2 probes and E2F1 probes were, respectively, incubated with cell extracts and streptavidin magnetic beads, with Bio-NC probes used as the controls. Finally, the enrichment of miR-184 was analyzed by RT-qPCR. Likewise, the specific probes for the Bio-ASK1 promoter were used and the enrichment of E2F1 was examined by RT-qPCR.

### 2.10. Fluorescence In Situ Hybridization (FISH) Assay

To study the location of circCNN2, FISH assays were performed using Fluorescent in Situ Hybridization Kits (C10910, RiboBio, Guangzhou, China) according to the manufacturer's requirements. DAPI was used to restain the nuclei. After that, Laser scanning confocal microscope (Smart zoom 5, Zeiss) was applied to observe the stained cells. GAPDH and U6 were treated as the cytoplasm and the nucleus control, respectively.

### 2.11. Chromatin Immunoprecipitation (ChIP) Assay

ChIP assay was implemented to testify the interplay between E2F1 and ASK1 promoter via using the ChIP assay kit (KT101-01, gzscbio, Gunagzhou, China). Cells were first cross-linked in 4% paraformaldehyde and then sonicated into chromatin fragments of 200-1000-bp which were incubated with the antibodies against E2F1 (ab4070, Abcam, UK) and negative control IgG (ab6789, Abcam, UK). After that, magnetic beads were added to enrich RNA, and finally, the immunoprecipitated RNAs were extracted and purified.

### 2.12. Luciferase Reporter Assay

To verify the binding capacity between E2F1 and ASK1 promoter, the sequence of ASK1 promoter was inserted into the downstream of pGL3 luciferase reporter vector to build pGL3-ASK1 promoter-Wt and pGL3- ASK1 promoter-Site1/2 Mut. The constructs were cotransfected with pcDNA3.1/E2F1 or pcDNA3.1 (control). All luciferase intensities were examined by luciferase reporter assay system (Promega) 36 hours after transfection and the binding sites between E2F1 and ASK1 promoter was verified.

For the verification of the binding capacity between circCNN2/E2F1 and miR-184, the full length of circCNN2 or E2F1 3′UTR possessing wild-type and mutant miR-184 binding sites were subcloned into pmirGLO luciferase vectors to obtain pmirGLO-circCNN2-Wt/Mut or pmirGLO-E2F1 3′UTR-Wt/Mut, which was then transfected with miR-184 mimics or mimics NC into LUSC cells. After 48-hour transfection, cells were extracted and the luciferase activities were analyzed utilizing the luciferase reporter assay system (Promega).

### 2.13. Subcutaneous Tumor Formation Experiment in Nude Mice

We referred related document and carried out the following animal experiments [16]. The male BALB/c nude mice (6-8-week-old) were acquired commercially from Shanghai Lab. Animal Research Center (Shanghai, China). Relevant animal experiments were carried out in accordance with the Animal Care and Use Committee guidelines of Tongji Hospital, Tongji Medical College, Huazhong University of Science and Technology. The mice were randomly divided into four groups (*n* = 6). After H1703 cells were transfected with sh1-circCNN2 (with sh-NC as the control) for 48 hours, 100 *μ*l of 2 × 10^7^ ml cells were obtained, and tumor volume was measured every three days as per the equation: *a* × *b*^2^ × 0.5 (*a*, long axes; *b*, short axes). After 28 days of injection, the mice were sacrificed and tumors were dissected for further detections.

### 2.14. Statistical Analysis

Each experiment was operated three times independently to ensure the accuracy of the results, and experimental data were demonstrated as the means ± SD. The statistical analysis, in form of Student's *t*-test or one-way ANOVA, was completed with application of SPSS 17.0 software. The two-sided *P* value less than 0.05 was considered to be statistically significant.

## 3. Results

### 3.1. circCNN2 Is Highly Expressed in LUSC Cells

According to UALCAN analysis, we found that CNN2, the host gene of circCNN2, was upregulated in LUSC tumor samples (Figure S1A). As previous study has elucidated that some circRNAs can be transcribed together with their parental genes and they in turn regulate the transcription of the parental gene [17], we speculated that circCNN2 may also exert potential role in LUSC progression, which led to the follow-up investigations. First, RT-qPCR was used to examine the expression of circCNN2 in LUSC cell lines (SK-MES-1, H1703, H226, and H520) and the normal human bronchial epithelial Beas-2B cell line (Figure 1(a)). The result showed that circCNN2 was highly expressed in LUSC cells, especially in H1703 and H226 cells. Therefore, these two cells were chosen for further studies, and three shRNAs targeting circCNN2 were designed and transfected into LUSC cells to reduce circCNN2 expression. RT-qPCR was conducted to examine the interference efficiency of circCNN2 in LUSC cells in H1703 and H226 cells (Figure S2A), and sh1-circCNN2 and sh2-circCNN2 with better transfection efficiency were selected for further studies. After that, the specific convergent and divergent primers were, respectively, designed to amplify circCNN2. The experimental data from gel electrophoresis displayed that circCNN2 was only amplified by cDNA templates instead of genomic DNA (gDNA) templates (Figure 1(b)). What is more, under the treatment of RNase R and Actinomycin D (Act D) with RT-qPCR to examine the expression of circCNN2 and CNN2, it was shown that CNN2 mRNA was significantly declined while no obvious change was seen in circCNN2 expression, and circCNN2 displayed a stabler structure than CNN2 after the Act D treatment (Figures 1(c) and 1(d)). The above data proved the loop structure as well as the stability of circCNN2. Before we explored the regulatory functions of circCNN2 on LUSC progression, FISH assay was carried out to identify the localization of circCNN2 in LUSC cells (Figure 1(e)), and the result showed that circCNN2 was mainly distributed in the cytoplasm of LUSC cells. In summary, circCNN2 expresses at a high level in LUSC cells.

### 3.2. circCNN2 Promotes Cell Proliferation and Invasion in LUSC

After we verified that circCNN2 was highly expressed in LUSC cells, we continued to explore the effects of circCNN2 silencing on the malignant phenotypes of LUSC cells. At first, CCK-8 and colony formation assays were conducted to examine the proliferative ability of H1703 and H226 cells after circCNN2 was knocked down (Figures 2(a) and 2(b)). The slower LUSC cell growth and reduced colony numbers demonstrated that circCNN2 silencing suppressed cell proliferation in LUSC. As proliferating cell nuclear antigen (PCNA) and cyclin D1 are important proliferation-associated proteins, we conducted western blot analysis to examine their protein levels in H1703 and H226 cells (Figure 2(c)). Results showed that the protein levels of PCNA and cyclin D1 were declined upon circCNN2 silencing. The above data indicated that circCNN2 silencing inhibited LUSC cell proliferation. Subsequently, Transwell assays were performed to analyze the effect of circCNN2 silencing on LUSC cell invasion (Figures 2(d) and 2(e)). Results showed that the invasive abilities of H1703 and H226 cells were reduced by circCNN2 downregulation. Likewise, western blot analysis was used to examine the protein levels of invasion-related proteins MMP2 and MMP9 in LUSC cells (Figure 2(f)), which showed that they were declined by circCNN2 knockdown. In summary, circCNN2 promotes LUSC cell proliferation and invasion.

### 3.3. circCNN2 Promotes LUSC Tumor Growth

After figuring out the regulatory role of circCNN2 in LUSC cell proliferation and invasion, we also designed several *in vivo* assays in nude mice to further verify the effect of circCNN2 on LUSC tumor growth. As shown in Figure 3(a), the growth rate of tumor volume in H1703 cells upon circCNN2 silencing was slower than that in the sh-NC group. Besides, it was shown from Figure 3(b) that tumor weight was decreased in the group transfecting with sh1-circCNN2. Besides, the expression of Ki67, the nuclear antigen representing cell proliferation, was analyzed by immunohistochemistry (Figure 3(c)). The result showed that the immunoreactivity and expression of Ki67 decreased after interference with circCNN2. Likewise, western blot analysis was utilized to examine the protein levels of proliferation-related proteins (PCNA and cyclin D1) and invasion-related proteins (MMP2 and MMP9) in different groups (Figure 3(d)). It was shown that the protein levels of the above proteins were decreased in the sh1-circCNN2 group compared with those in the sh-NC group. In a word, circCNN2 facilitates LUSC tumor growth.

### 3.4. circCNN2 Functions as a ceRNA by Competitively Sponging miR-184

Since FISH assay in Figure 1(e) suggested that circCNN2 was mainly distributed in the cytoplasm of LUSC cells, we speculated that circCNN2 may exert its functions in LUSC as a ceRNA. We adopted RIP assay with gel electrophoresis to detect the enrichment of circCNN2 in RNA-induced silencing complex (RISC) (Figures 4(a) and 4(b)). It was found that circCNN2 was enriched in the anti-AGO2 group compared with the anti-IgG group, suggesting the potential ceRNA network of circCNN2 in LUSC cells. Next, we applied the starBase (http://starbase.sysu.edu.cn) database to predict potential miRNAs that could bind to circCNN2, and miR-184 was found to be the candidate (Figure S2B). Since previous studies have elucidated that miR-184 was downregulated in lung cancer [18–20], we chose to investigate it in the next-step studies. RT-qPCR was used to examine the expression of miR-184 in H1703 and H226 cells compared with that in the Beas-2B cell line (Figure 4(c)). Results showed that miR-184 was downregulated in LUSC cells. Then, the transfection efficiency of miR-184 was examined via RT-qPCR (Figure S2C-D). It was observed through RIP assay that miR-184 was also enriched in the anti-AGO2 group, indicating the binding capacity between miR-184 and circCNN2 (Figure 4(d)). After that, RNA pull down assay was carried out to detect miR-184 enrichment in different groups, and results showed that miR-184 was obviously enriched in the Bio-circCNN2-Wt group while the mutated group displayed no obvious change (Figure 4(e)). Results of luciferase reporter assay indicated that the luciferase activity of LUSC cells in the pmirGLO-circCNN2-Wt group was declined by miR-184 mimics while the mutated group displayed no significant change (Figure 4(f)). The above data indicated the binding ability between circCNN2 and miR-184. Furthermore, RT-qPCR was conducted to examine miR-184 expression in H1703 and H226 cells after inhibiting circCNN2 (Figure 4(g)). The result showed that circCNN2 could bind to miR-184 without affecting its expression, which further proved the ceRNA role of circCNN2 in LUSC cells. What is more, the effects of circCNN2/miR-184 on LUSC progression were explored by a series of rescue assays. Results from CCK-8 and colony formation assays showed that the suppressed LUSC cell proliferation caused by circCNN2 knockdown was reversed by the cotransfection of miR-184 inhibitor (Figure S3A-B). Western blot was conducted to detect the protein changes of proliferation-related proteins in different transfection groups, and results showed that declined PCNA and cyclin D1 protein levels caused by circCNN2 silencing was countervailed by miR-184 inhibition (Figure S3C). In addition, results of Transwell assays demonstrated that the silencing of miR-184 could reverse the inhibitory effect of circCNN2 downregulation on LUSC cell invasion, and the protein levels of invasion-related factors detected via western blot analysis showed same results (Figure S3D-F). In a word, circCNN2 competitively sponges miR-184 in LUSC cells.

### 3.5. circCNN2 Upregulates E2F1 Expression via miR-184

For next-step study, we applied the starBase database (selection condition: high stringency (≥3), 10 cancer types) to predict the potential downstream mRNAs of miR-184. As shown in Figure S4A, eight mRNAs (H2AFX, LSM4, ARHGAP39, CLUH, MDH2, E2F1, CDCA4, and TIMM13) were selected as candidates. After that, RT-qPCR was used to examine the expression of the above mRNAs upon circCNN2 knockdown (Figure 5(a)). Results showed that only E2F1 was prominently declined by sh-circCNN2. Therefore, we chose E2F1 for further investigations. It was shown through RT-qPCR and western blot that the expression and protein levels of E2F1 were reduced by circCNN2 knockdown (Figures 5(b) and 5(c)). Subsequently, we used RT-qPCR and western blot to examine E2F1 expression and protein levels in H1703 and H226 cells, and results showed that E2F1 was upregulated in LUSC cells (Figure 5(d)). The transfection efficiency of E2F1 was examined via RT-qPCR, and sh1/2-E2F1 was selected for further studies (Figure S4B-C). After that, RT-qPCR and western blot assays were conducted to detect the expression and protein levels of E2F1 upon miR-184 inhibition, which showed a negative regulation between E2F1 and miR-184 (Figure 5(e)). It was verified by RNA pull down assay that the wild type of biotinylated E2F1 probe could pull down miR-184 while no obvious change was seen in the mutated group (Figure 5(f)). Likewise, it was observed through luciferase report assay that the luciferase activity of LUSC cells was declined in pmirGLO-E2F1 3′UTR-Wt groups rather than in the mutated group (Figure 5(g)). The above data demonstrated the binding ability between E2F1 and miR-184. Finally, a series of rescue assays were conducted to verify the regulatory mechanism among circCNN2, miR-184 and E2F1. As shown in Figure 5(h), the expression and protein levels of E2F1 were declined by circCNN2 silencing, while such effect was reversed by the cotransfection of the miR-184-inhibitor. All in all, circCNN2 upregulates E2F1 expression by competitively binding to miR-184. Furthermore, the effects of miR-184/E2F1 on LUSC progression were explored by rescue assays. It was observed through CCK-8 and colony formation assays that the repressed LUSC cell proliferation caused by overexpressing miR-184 was countervailed by the cotransfection of pcDNA3.1-E2F1 (Figure S5A-B). Besides, as shown in Figure S5C, the declined protein levels of proliferation-related proteins caused by miR-184 overexpression was counteracted by E2F1 upregulation. Subsequently, Transwell assays were carried out to detect cell invasion upon different transfection conditions, and results demonstrated that the up-regulation of E2F1 reversed the inhibitory effect of miR-184 overexpression on LUSC cell invasion (Figure S5D-E). It was also shown in Figure S5F that increased E2F1 expression counteracted the reduced invasion-related protein levels caused by miR-184 overexpression. In a word, circCNN2 up-regulates E2F1 expression via miR-184 in LUSC cells.

### 3.6. circCNN2 Activates MAPK Signaling Pathway by Upregulating ASK1 Expression via E2F1

Experimental data from early reports illustrates that E2F1 transcriptionally activates apoptosis signal-regulating kinase 1 (ASK1) [21], and ASK1 serves as a regulator of MAPK signaling pathway [22, 23]. Next, we decided to verify whether circCNN2 could regulate the MAPK signaling pathway by transcriptionally activating ASK1 expression through E2F1 in LUSC. Firstly, RT-qPCR and western blot assays were conducted to examine the expression and protein levels of ASK1 in H1703 and H226 cells, and it was shown that ASK1 was up-regulated in LUSC cells (Figure 6(a)). It was then observed through RT-qPCR and western blot analysis that the expression and protein levels of ASK1 was declined by E2F1 silencing in H1703 and H226 cells (Figures 6(b) and 6(c)). Subsequently, results of ChIP and DNA pull down assay showed that the ASK1 promoter was enriched in the anti-E2F1 groups, and the biotinylated ASK1 promoter could pull down E2F1 antibody (Figures 6(d) and 6(e)). The above data demonstrated the binding ability between E2F1 and the ASK1 promoter. For the next step, we applied the JASPAR (http://jaspar.genereg.net/) database to predict the binding sites between E2F1 and ASK1 promoter (Figure S6A), and then, site#1 and site#2 with the highest reliability (score > 10) were selected for subsequent experiments. Luciferase reporter assay was then conducted to identify the specific binding site, and results showed that the luciferase activity of LUSC cells was only declined after site 1 was mutated, which indicated that E2F1 bound to the ASK1 promoter at site 1 (Figure 6(f)). Next, we explored the regulatory effect of E2F1 on the MAPK signaling pathway. As p38 is a key protein in the regulation of the MAPK signaling pathway, we conducted western blot analysis to examine its protein level in LUSC cells upon E2F1 downregulation (Figure 6(g)). Results showed that after silencing E2F1, the protein level of p38 remained unchanged while its phosphorylation level (p-p38) decreased, indicating that the MAPK signaling pathway was inhibited. After that, RT-qPCR and western blot assay were conducted to examine the expression and protein levels of ASK1 under different transfection conditions (Figures 6(h) and 6(i)). Results showed that after silencing circCNN2, ASK1 expression and protein levels declined, while this effect was reversed by overexpressing E2F1. It was also observed through western blot analysis that the decreased protein level of p-p38 caused by circCNN2 knockdown was recovered by the cotransfection of pcDNA3.1-E2F1. The above data demonstrated that circCNN2 transcriptionally elevating ASK1 expression through E2F1 and thus activating the MAPK signaling pathway in LUSC.

## 4. Discussion

As a major subtype of lung cancer, LUSC is associated with poor clinical prognosis and lacks available targeted therapy. Therefore, it is necessary to provide novel molecular targets for the treatment of LUSC [3]. In this study, we found that the host gene of circCNN2 was upregulated in LUSC tumor samples, so we speculated that circCNN2 may exert regulatory functions in LUSC. We firstly verified the high expression pattern of circCNN2 as well as its stable circular structure in LUSC cells. Then, with the application of functional assays and animal studies, circCNN2 was verified to promote LUSC cell proliferation and invasion *in vitro* and promote LUSC tumor growth *in vivo*. These findings identified circCNN2 as a potential biomarker which may exert therapeutic options for the treatment of LUSC.

The ceRNA network involving lncRNAs, circRNAs, and miRNAs in the regulation of cancer development has been validated by many studies, in which lncRNAs/circRNAs may act as ceRNAs by competitively binding to miRNAs to regulate the expression levels of miRNA target mRNAs [24]. Importantly, the function of circRNAs in cancer cells has been illustrated, including in LUSC [25, 26]. In the present research, it was observed through FISH assay that circCNN2 was mainly located in the cytoplasm of LUSC cells, which suggested the possibility of the ceRNA pattern. With the help of informatics prediction and mechanism experiments, it was verified that circCNN2 could bind to miR-184 and E2F1 was the target mRNA of miR-184 in LUSC cells. Besides, it was verified that circCNN2 facilitated LUSC cell proliferation and invasion by binding to miR-184 to enhance E2F1. miR-184 has been largely reported to be involved in a variety of cancers, in which it exerts oncogenic or anti-tumor impact on cell progression [18]. For example, miR-184 inhibits cell proliferation and invasion in glioma [27] and suppresses neuroblastoma cell survival [28], while it functions as potential oncogenic miRNA of squamous cell carcinoma of tongue [29]. Consistent with the previous findings, we found in this study that miR-184 was downregulated in LUSC cells, which made it a potential biomarker for LUSC treatment.

The MAPK signaling pathway has been reported to be associated with cell proliferation, migration and apoptosis [12]. What is more, the MAPK signaling pathway has been reported to exert crucial functions in the development of lung cancer [12, 30]. By referring to related documents, we found that E2F1 can transcriptionally activate ASK1 [21], and ASK1 can serve as an activation regulator of the MAPK signaling pathway [22, 23]. Therefore, we decided to verify the interaction among circCNN2, E2F1, and ASK1 in the MAPK signaling pathway. We first identified the binding ability between the E2F1 and ASK1 promoters, and then, we found through a series mechanism experiments that circCNN2 could transcriptionally elevate ASK1 expression through E2F1 and thus activating the MAPK signaling pathway in LUSC. These findings indicated that circCNN2 may have regulatory function on the activation of the MAPK signaling pathway, which may help offer effective therapeutic strategies for LUSC in the future.

## 5. Conclusion

Our study indicates that circCNN2 activates the MAPK signaling pathway via the miR-184/E2F1 axis, thereby promoting LUSC cell proliferation and invasion. Though more efforts are still needed to be made to support the clinical significance of circCNN2 in the researches on LUSC, we hope that this study may help to shed novel insights on the treatment of LUSC in the future.

## Figures and Tables

**Figure 1:** circCNN2 is highly expressed in LUSC cells. (a) RT-qPCR was used to examine the expression of circCNN2 in LUSC cell lines (SK-MES-1, H1703, H226, and H520) and the normal human bronchial epithelial Beas-2B cell line. (b) The specific convergent and divergent primers were, respectively, designed to amplify circCNN2, and gel electrophoresis with RT-qPCR was conducted to verify the loop structure of circCNN2. (c, d) RNase R and Actinomycin D (Act D) was used to treat H1703 and H226 cells and RT-qPCR was used to examine the expression of circCNN2 and CNN2. (e) FISH assay was carried out to identify the localization of circCNN2 in LUSC cells. ^∗^*P* < 0.05, ^∗∗^*P* < 0.01 compared to the control group.

**Figure 2:** circCNN2 promotes cell proliferation and invasion in LUSC. (a, b) CCK-8 and colony formation assays were conducted to evaluate the proliferative ability of H1703 and H226 cells after circCNN2 was silenced. (c) Western blot analysis was performed to examine the protein levels of PCNA and cyclin D1 in H1703 and H226 cells upon circCNN2 silencing. (d, e) Transwell assays were performed to analyze the effect of circCNN2 silencing on LUSC cell invasion. (f) Western blot analysis was used to examine the protein levels of invasion-related proteins MMP2 and MMP9 in LUSC cells. ^∗∗^*P* < 0.01 compared to the sh-NC group.

**Figure 3:** circCNN2 promotes LUSC tumor growth. (a) The tumor volume in H1703 cells upon circCNN2 knockdown was examined via RT-qPCR. (b) Tumor weight in H1703 cells upon circCNN2 silencing was measured via RT-qPCR. (c) The expression of Ki67, the nuclear antigen representing cell proliferation, was analyzed by immunohistochemistry. (d) Western blot analysis was utilized to examine the protein levels of proliferation-related proteins (PCNA and cyclin D1) and invasion-related proteins (MMP2 and MMP9) in different tumor groups. ^∗∗^*P* < 0.01 compared to the sh-NC group.

**Figure 4:** circCNN2 functions as a ceRNA by competitively sponging miR-184. (a, b) RIP assay with gel electrophoresis was conducted to detect the enrichment of circCNN2 in RNA-induced silencing complex (RISC). (c) RT-qPCR was used to examine the expression of miR-184 in H1703 and H226 cells compared with Beas-2B cell line. (d) RIP assay was carried out to evaluate miR-184 enrichment in anti-AGO2 and anti-IgG groups. (e) RNA pull down assay was adopted to test the enrichment of miR-184 in Bio-circCNN2-Wt and Bio-circCNN2-Wut groups. (f) Luciferase report assays were conducted to evaluate the luciferase activity of wild-type or mutant circCNN2 plasmids upon mimics NC and miR-184 mimics. (g) RT-qPCR was conducted to examine miR-184 expression in H1703 and H226 cells after inhibiting circCNN2. ^∗∗^*P* < 0.01 compared to the control group.

**Figure 5:** circCNN2 upregulates E2F1 expression via miR-184. (a) RT-qPCR was used to examine the expression of 8 candidate mRNAs (H2AFX, LSM4, ARHGAP39, CLUH, MDH2, E2F1, CDCA4, and TIMM13) upon circCNN2 knockdown. (b, c) RT-qPCR and western blot assays were conducted to test the expression and protein levels of E2F1 upon circCNN2 knockdown in H1703 and H226 cells. (d) RT-qPCR and western blot analysis were used to examine the expression and protein levels of E2F1 in LUSC cells. (e) RT-qPCR and western blot assays were conducted to detect the expression and protein levels of E2F1 upon miR-184 downregulation. (f) RNA pull down assay was carried out to verify the binding ability between miR-184 and E2F1 with Bio-NC as the control. (g) The binding ability between miR-184 and E2F1 was verified through luciferase report assay by testing the luciferase activity of LUSC cells transfected with wild-type or mutated E2F1 plasmids upon mimics NC and miR-184 mimics. (h) Rescue assays were conducted to verify the interaction among circCNN2, miR-184 and E2F1. ^∗∗^*P* < 0.01 compared to the control group.

**Figure 6:** circCNN2 activates MAPK signaling pathway by upregulating ASK1 expression via E2F1. (a) RT-qPCR and western blot assays were conducted to examine the expression and protein levels of ASK1 in LUSC cells. (b, c) RT-qPCR and western blot analysis were used to examine the expression and protein levels of ASK1 after E2F1 was knocked down in H1703 and H226 cells. (d, e) ChIP and DNA pull down assay were carried out to verify the binding ability between E2F1 and ASK1 promoter. (f) Luciferase reporter assay was conducted to detect the specific binding site between E2F1 and ASK1 promoter. (g) Western blot was conducted to detect the protein levels of p38 and p-p38 upon E2F1 silencing. (h) RT-qPCR was used to examine the expression of ASK1 in different transfection groups. (i) Western blot assay was conducted to examine the protein levels of p38, p-p38, and ASK1 under different transfection conditions. ^∗∗^*P* < 0.01 compared to the control group.

## Data Availability

Data will be available upon reasonable requests from the corresponding author.

## Supplementary Materials

Supplementary Materials Figure S1: (A) the expression of CNN2, the host gene of circCNN2 in LUSC tumor samples was predicted through UALCAN analysis. Figure S2: (A) the interference efficiency of circCNN2 in H1703 and H226 cells was detected by RT-qPCR. (B) StarBase database was used to predict potential miRNAs that could bind to circCNN2. (C) RT-qPCR was used to examine the overexpression efficiency of miR-184 in H1703 and H226 cells. (D) RT-qPCR was used to examine the interference efficiency of miR-184 in H1703 and H226 cells. ^∗∗^*P* < 0.01 compared to the control group. Figure S3: a series of rescue assays were conducted to examine the effects of circCNN2/miR-184 on LUSC cell proliferation and invasion. Experimental groups were divided into sh-NC, sh1-circCNN2, sh1-circCNN2+inhibitor NC, and sh1-circCNN2+miR-184 inhibitor. (A-B) CCK-8 and colony formation assays were conducted to examine the proliferative ability of H1703 and H226 cells in different groups. (C) Western blot analysis was utilized to examine the protein levels of PCNA and cyclin D1 in different groups. (D-E) Transwell assays were performed in different groups to analyze the effect of circCNN2 silencing on LUSC cell invasion. (F) Western blot analysis was used to examine the protein levels of invasion-related proteins MMP2 and MMP9 in LUSC cells under different conditions. ^∗∗^*P* < 0.01 compared to the control group. Figure S4: (A) potential mRNAs that could bind to miR-184 were predicted through starBase database. (B) The interference efficiency of E2F1 in H1703 and H226 cells was detected by RT-qPCR. (C) RT-qPCR was used to examine the overexpression efficiency of E2F1 in LUSC cells. ^∗∗^*P* < 0.01 compared to the control group. Figure S5: a series of rescue assays were conducted to examine the effects of miR-184/E2F1 on LUSC cell proliferation and invasion in different groups transfected with mimics-NC, miR-184 mimics, miR-184+pcDNA3.1, and miR-184 mimics+pcDNA3.1-E2F1 plasmids. (A, B) CCK-8 and colony formation assays were conducted to examine the proliferative ability of H1703 and H226 cells in different groups. (C) Western blot analysis to examine the protein levels of PCNA and cyclin D1 in H1703 and H226 cells under different conditions. (D, E) Transwell assays were performed to analyze the effect of circCNN2 silencing on LUSC cell invasion. (F) Western blot analysis was used to examine the protein levels of invasion-related proteins MMP2 and MMP9 in LUSC cells under different conditions. ^∗∗^*P* < 0.01 compared to control group. Figure S6 The binding sites between E2F1 and ASK1 promoters were predicted through JASPAR database.

## References

[1] Schwartz A. G., Cote M. L. (2016). Epidemiology of lung cancer. *Advances in Experimental Medicine and Biology*.

[2] Bezzecchi E., Ronzio M., Dolfini D., Mantovani R. (2019). NF-YA Overexpression in lung cancer: LUSC. *Genes*.

[3] Li Y., Gu J., Xu F., Zhu Q., Ge D., Lu C. (2018). Transcriptomic and functional network features of lung squamous cell carcinoma through integrative analysis of GEO and TCGA data. *Scientific Reports*.

[4] Kristensen L. S., Andersen M. S., Stagsted L. V. W., Ebbesen K. K., Hansen T. B., Kjems J. (2019). The biogenesis, biology and characterization of circular RNAs. *Nature Reviews. Genetics*.

[5] Chen L., Nan A., Zhang N. (2019). Circular RNA 100146 functions as an oncogene through direct binding to miR-361-3p and miR-615-5p in non-small cell lung cancer. *Molecular Cancer*.

[6] Zhang N., Nan A., Chen L. (2020). Circular RNA circSATB2 promotes progression of non-small cell lung cancer cells. *Molecular Cancer*.

[7] Wang C., Tan S., Liu W. R. (2019). RNA-Seq profiling of circular RNA in human lung adenocarcinoma and squamous cell carcinoma. *Molecular Cancer*.

[8] Zeng K., Chen X., Xu M. (2018). CircHIPK3 promotes colorectal cancer growth and metastasis by sponging miR-7. *Cell Death & Disease*.

[9] Yu J., Yang M., Zhou B. (2019). CircRNA-104718 acts as competing endogenous RNA and promotes hepatocellular carcinoma progression through microRNA-218-5p/TXNDC5 signaling pathway. *Clinical Science (London, England)*.

[10] Cheng Z., Yu C., Cui S. (2019). circTP63 functions as a ceRNA to promote lung squamous cell carcinoma progression by upregulating FOXM1. *Nature Communications*.

[11] Zhang W., Shi J., Cheng C., Wang H. (2020). CircTIMELESS regulates the proliferation and invasion of lung squamous cell carcinoma cells via the miR-136-5p/ROCK1 axis. *Journal of Cellular Physiology*.

[12] Sun Y., Liu W. Z., Liu T., Feng X., Yang N., Zhou H. F. (2015). Signaling pathway of MAPK/ERK in cell proliferation, differentiation, migration, senescence and apoptosis. *Journal of Receptor and Signal Transduction Research*.

[13] Soleimani A., Rahmani F., Saeedi N. (2019). The potential role of regulatory microRNAs of RAS/MAPK signaling pathway in the pathogenesis of colorectal cancer. *Journal of Cellular Biochemistry*.

[14] Burotto M., Chiou V. L., Lee J. M., Kohn E. C. (2014). The MAPK pathway across different malignancies: a new perspective. *Cancer*.

[15] Guo L., Li B., Yang J., Shen J., Ji J., Miao M. (2020). Fibroblast-derived exosomal microRNA-369 potentiates migration and invasion of lung squamous cell carcinoma cells via NF1-mediated MAPK signaling pathway. *International Journal of Molecular Medicine*.

[16] Tian X., Wu Y., Yang Y. (2020). Long noncoding RNA LINC00662 promotes M2 macrophage polarization and hepatocellular carcinoma progression via activating Wnt/*β*-catenin signaling. *Molecular Oncology*.

[17] Qi J. C., Yang Z., Lin T. (2021). CDK13 upregulation-induced formation of the positive feedback loop among circCDK13, miR-212-5p/miR-449a and E2F5 contributes to prostate carcinogenesis. *Journal of Experimental & Clinical Cancer Research*.

[18] Tung M. C., Lin P. L., Cheng Y. W. (2016). Reduction of microRNA-184 by E6 oncoprotein confers cisplatin resistance in lung cancer via increasing Bcl-2. *Oncotarget*.

[19] Wu L., Liu C., Zhang Z. (2020). Knockdown of lncRNA MIAT inhibits proliferation and cisplatin resistance in non-small cell lung cancer cells by increasing miR-184 expression. *Oncology Letters*.

[20] Ding H., Wen W., Ding Q., Zhao X. (2020). Diagnostic valuation of serum miR-184 and miR-191 in patients with non-small-cell lung cancer. *Cancer Control*.

[21] Haim Y., Blüher M., Konrad D. (2017). ASK1 (MAP3K5) is transcriptionally upregulated by E2F1 in adipose tissue in obesity, molecularly defining a human dys-metabolic obese phenotype. *Mol Metab*.

[22] Liu T., Lin J., Chen C. (2021). MicroRNA-146b-5p overexpression attenuates premature ovarian failure in mice by inhibiting the Dab2ip/Ask1/p38-Mapk pathway and *γ*H2A.X phosphorylation. *Cell Proliferation*.

[23] Meijles D. N., Cull J. J., Markou T. (2020). Redox regulation of cardiac ASK1 (apoptosis signal-regulating kinase 1) controls p38-MAPK (mitogen-activated protein kinase) and orchestrates cardiac remodeling to hypertension. *Hypertension*.

[24] Zhu J., Zhang X., Gao W., Hu H., Wang X., Hao D. (2019). lncRNA/circRNA-miRNA-mRNA ceRNA network in lumbar intervertebral disc degeneration. *Molecular Medicine Reports*.

[25] Yu M., Tian Y., Wu M. (2020). A comparison of mRNA and circRNA expression between squamous cell carcinoma and adenocarcinoma of the lungs. *Genetics and Molecular Biology*.

[26] Wang Y., Zhang H., Wang J., Li B., Wang X. (2020). Circular RNA expression profile of lung squamous cell carcinoma: identification of potential biomarkers and therapeutic targets. *Bioscience Reports*.

[27] Cheng Z., Wang H. Z., Li X. (2015). MicroRNA-184 inhibits cell proliferation and invasion, and specifically targets TNFAIP2 in glioma. *Journal of Experimental & Clinical Cancer Research*.

[28] Foley N. H., Bray I. M., Tivnan A. (2010). MicroRNA-184 inhibits neuroblastoma cell survival through targeting the serine/threonine kinase AKT2. *Molecular Cancer*.

[29] Wong T. S., Liu X. B., Wong B. Y. H., Ng R. W. M., Yuen A. P. W., Wei W. I. (2008). Mature miR-184 as potential oncogenic microRNA of squamous cell carcinoma of tongue. *Clinical Cancer Research*.

[30] Zhou Z., Zhou Q., Wu X. (2020). VCAM-1 secreted from cancer-associated fibroblasts enhances the growth and invasion of lung cancer cells through AKT and MAPK signaling. *Cancer Letters*.

